The article "A Biomechanical Study on Failed Snatch Based on the Human and Bar Combination Barycenter" was published in 2022. Journal: Appl Bionics Biomech.

# A Biomechanical Study on Failed Snatch Based on the Human and Bar Combination Barycenter

**DOI:** 10.1155/2022/9279638

**Published:** 2022-05-10

**Authors:** Gongju Liu, Houwei Zhu, Jing Ma, Huiju Pan, Xu Pan, Yingyue Zhang, Ting Hu, Gusztáv Fekete, Haiying Guo, Minjun Liang

**Affiliations:** ^1^Scientific Research Department, Zhejiang College of Sports, China; ^2^Faculty of Engineering, University of Pannonia, Hungary; ^3^College of Physical Education and Health Sciences, Zhejiang Normal University, China; ^4^Research Academy of Grand Health, Ningbo University, China; ^5^Department of Physical and Health Education, Udon Thani Rajabhat University, Thailand

## Abstract

**Objective:**

The purpose of this research was to use a new method the human and bar combination barycenter to exposit the differences between successful and failed characteristics of snatch attempts in competition. Try to establish an effective biomechanical method that can uncover the main factors for the failed snatch. The obtained results will provide valuable information for weightlifters to improve the success rate in snatch by altering their technical issues accordingly.

**Methods:**

A 3-D video analysis method was used to compare the characteristics of the heaviest successful and failed attempts of ten elite weightlifters in the men's 73 kg category. The video was captured under competitive conditions at the 2019 World Weightlifting Championships, the 2019 Asian Weightlifting Championships, and the 2020 China Olympic Trial. The video data were digitized using the SIMI°Motion7.50 3-D system (Germany).

**Results:**

Significant difference (*P* > 0.05) was not found between the successful and failed attempts in the parameters, such as the maximal vertical rising velocity, the maximal vertical height, and the vertical displacement of the barbell. The maximal descending acceleration of the human body, the time duration, the angles of the hip, and knee joints were no significant difference. However, significant differences were found in the variation of the human and bar combination barycenter on the *X-*axis in the inertial ascent stage and the squat support stage (*t* = 2.862, *P* < 0.05; *t* = 3.376, *P* < 0.05).

**Conclusions:**

A probable cause of the failed snatch is that the displacement of human and bar combination barycenter on the *X-*axis is not enough to reach the position for supporting barbell during the inertial ascent stage and the squat support stage. The reason is that the strength of reclining of torso at the end of the force phase is insufficient. Insufficient knee flexion in the knee flexion phase (*M*2), which leads to a lower maximum vertical velocity of barbell, may be an indirect factor leading to the failed snatch. The cumulative variation of human and bar combination barycenter on the *X-*axis can effectively determine the technical characteristics between the success and failure in snatch.

The article "A Biomechanical Study on Failed Snatch Based on the Human and Bar Combination Barycenter" was published in 2022. Journal: Appl Bionics Biomech.

## 1. Introduction

The technical principle of the snatch shows that weightlifters need to follow the three principles of “Near,” “Fast,” and “Low” during the snatch process [1, 2]. “Near” means that the barbell is required to be as close to the body as possible during the lifting, which is determined by the horizontal distance (*L*_*H*_) between the center of gravity (COG) of barbell and human body [3]. “Fast” means that pulling the barbell and action force should be fast, which is determined by the maximal velocity at the end of the force phase (*V*_max_) [3]. “Low” refers to requiring lifters to reduce the *COG* of body at the fastest speed to facilitate the support to the barbell, which is determined by the biggest falling acceleration (*a*_*f*_) of *COG* of body during the squat support stage [3].

With the application of 3-D technology, the parameters which were used to determine the three principles are more diverse and precise. The maximal height (*H*_bmax_) and the fall distance of the barbell (*H*_bd_) are the key parameters to evaluate the support technique [4, 5]. The trajectory of *COG* of barbell and body are used as an overall analysis of snatch technical characteristics [6–8]. Spatial-temporal characteristics and angle of joints of human body are parameters for evaluating the structure of the snatch after the division of snatch movement [9, 10]. Phases of snatch reveal that the snatch technique must not only conform to the mechanics principle but also adapt to the body structure and physiological characteristics. “Phases” of snatch is an important supplement to the three principles, which can be called the fourth principle.

In recent years, there are many studies on the technical characteristics of elite weightlifters in terms of snatch structure evaluation, *COG* of barbell, and *COG* of human body. Wang et al. and Li et al. used 3-D kinematics method to analyze the time structure, the changes of barbell space structure, and joints angle characteristics of different phases of Chinese female elite weightlifters [9, 10]. Yang et al. and Erbil compared the technical differences between male and female lifters in a series parameters such as time structure, barbell spatial structure, work ratio, and joints angle [11, 12]. Ikeda et al. and Musser et al. analyzed the technical differences among different categories [13, 14]. Some studies compared the successful and unsuccessful snatch technique of elite lifters in temporal structure, spatial structure, and characteristics of *COG* of barbell in phases [15–17].

The article "A Biomechanical Study on Failed Snatch Based on the Human and Bar Combination Barycenter" was published in 2022. Journal: Appl Bionics Biomech.

Wang et al. reported that the failed snatch of most elite lifters occurred during the support completion phase [18]. Therefore, it is speculated that the main reason for failure of forward or backward is that the position of the *COG* of human body and barbell on the sagittal plan exceeds the lifters' control limit. Since the trajectory of the *COG* of barbell will be different of every attempt of each lifter, there is a certain relationship between the trajectories of the *COG* of barbell and human body. Therefore, it is difficult to find the difference between successful and failed attempts only from the trajectory of the *COG* of human body or barbell. In this case, the human and bar combination barycenter may be a good choice. The concept of human and bar combination barycenter was first coined by Wang in 1984 [19], due to the technical limitations, the characteristics and the roles of human and bar combination barycenter were not explained in their research at that time. Although there are some studies that try to compare successful and failed attempts, this is insufficient and the factors of failed snatch are still unclear.

In the snatch competition, each athlete only has 3 attempts to lift the barbell, so the success rate is the guarantee for the best results. The present study proposes to use the human and bar combination barycenter as the parameter to compare the successful and failed snatch attempts. The purpose of the present research is to analyze the three principles of “Near,” “Fast,” and “Low,” the phased principle, and the human and bar combination barycenter, to exposit the differences between successful and failed characteristics of snatch in competition, and to explore the biomechanical factors that cause the snatch failure.

## 2. Subjects and Methods

### 2.1. Subjects

The data were captured in the final A of World Weightlifting Championships (2019), the Asian Weightlifting Championships (2019), and the China Olympic Trial (2020). The weightlifters in the men's 73 kg category of snatch competition were selected, and the attempts of their maximum weights for success and failure were selected for analysis. The selection criteria for the unsuccessful performances are that the moment of failure must occur in the support completion phase, and all the unsuccessful performances are forward falling to facilitate the data analysis. Data on height, body mass, and maximum successful and failed results are shown in Table 1. The present study was authorized by the Ethics Committee of General Administration of Sport of China. All video data are from public competitions, and the video collection method used will not affect the athletes' performance in any way.

The article "A Biomechanical Study on Failed Snatch Based on the Human and Bar Combination Barycenter" was published in 2022. Journal: Appl Bionics Biomech.

### 2.2. Experimental Design

#### 2.2.1. Camera System and Coordinate System

*(1) Camera System*. In order to acquire kinematic indexes of human body and barbell, according to the on-site surroundings, we used two professional cameras, which were set approximately 15 meters from the center of the platform. The optical axis of the two cameras formed an angle of about 45° with the middle line of frontal plane (Figure 1(a)). The focal length and position of the two cameras kept unchanged during the whole competition. The raw data were smoothed using a low-pass digital filter with the 4 Hz of cut-off frequency [11, 20].

*(2) Coordinate System*. One hour before the snatch competition starts, we used the PEAK 3-D framework to calibrate the space of weightlifting platform (Figure 1(b)). At the beginning of snatch, the coordinates of the *COG* of barbell are set to (0, 0, and 22.5) in cm, and the coordinates of position of human body and barbell correspond to it during the movement. The setting of coordinate system is that the positive direction of *X-*axis is directly behind the lifter, the positive direction of *y-*axis is on the right side, and the positive direction of *Z-*axis is vertically upward (Figure 1(c)).

#### 2.2.2. Data Collection and Calculation

*(1) Phases Division of Snatch*. The snatch process was divided into six phases in most previous studies; they are the first pull phase, the transition phase, the second pull phase, the turnover phase, the catch phase, and fully stand phase [11, 21–24]. And they reported that the phases before the full stand were the most important in snatch [20, 22, 25, 26]. In the present study, the snatch action from start to end of squat position, which is consistent with literature, was divided as the knee extension phase, the knee flexion phase, the force phase, the inertial ascent phase, the squat support phase, and the support completion phase, which were abbreviated as *M*1-*M*6 [27]. The characteristics of each phase are shown in Figure 2; each picture represents the beginning and end of the phase.

*(2) Data Collection*. In order to calculate the kinematic indexes of human body and barbell, seventeen key points were manually digitized in the SIMI°Motion7.50 3-D system (Figure 3). These key points include the head, bilateral shoulder, bilateral elbow, bilateral wrist, bilateral hip, bilateral knee, bilateral ankle bone, bilateral tiptoe, and two endpoints of barbell [28]. The *COG* position of barbell was calculated form the geometric center of the two endpoints of barbell, and the *COG* position of human body was obtained by Hanavan Body Mathematical Model; they were obtained in the SIMI°Motion system automatically.

The article "A Biomechanical Study on Failed Snatch Based on the Human and Bar Combination Barycenter" was published in 2022. Journal: Appl Bionics Biomech.

In the present study, several variables were selected to assess the three principles of “Near,” “Fast,” and “Low” and the characteristics of phases. The minimum horizontal distance between the *COG* of barbell and human body when the barbell was rising (*L*_Hmin_) was selected for assessing the “Near” principle. The maximal vertical rising velocity (*V*_max_) and the maximal vertical height of barbell (*H*_bmax_) were selected to assess the “Fast” principle [16]. At the end of *M*3, the lifter's body begins to squat down quickly, at which time the maximum falling acceleration of the *COG* of body (*a*_*f*_), the vertical distance between the *COG* of barbell and human body at the end of *M*4 (*L*_Hz1_) and *M*5 (*L*_Hz2_), and the vertical height of human body (*H*_bd5_) and barbell (*H*_b5_) at the end of *M*5 were selected for assessing the “Low” principle. The vertical displacement of barbell and the time duration of each phase and the angles of hip and knee joints at the end of each phase were chosen to assess the characteristics of phases.

*(3) Human and Bar Combination Barycenter Calculation*. The original coordinate data of *COG* of barbell and human body were exported by the SIMI°Motion system, and the position of human and bar combination barycenter was calculated by the following formulas.

*(4) Calculation of *X*-Axis Coordinates of Human and Bar Combination Barycenter (*X*_*c*_)*. The *COG* of human body position on the *X-*axis is *X*1, the *COG* of barbell position on the *X-*axis is *X*2, the weight of lifter is *M*1, and the weight of barbell is *M*2.

(1) $$\begin{array}{c} X_{c}=\frac{\left(X1\times M1+X2\times M2\right)}{\left(M1+M2\right)}. \end{array}$$

*(5) Calculation of *Y*-Axis Coordinates of Human and Bar Combination Barycenter (*Y*_*c*_)*. The *COG* of human body position on the *Y-*axis is *Y*1, the *COG* of barbell position on the *Y-*axis is *Y*2, the weight of lifter is *M*1, and the weight of barbell is *M*2.

(2) $$\begin{array}{c} Y_{c}=\frac{\left(\text{Y}1\times M1+Y2\times M2\right)}{\left(M1+M2\right)}. \end{array}$$

*(6) Calculation of Z-Axis Coordinates of Human and Bar Combination Barycenter (*Z*_*c*_)*. The *COG* of human body position on the *Z-*axis is *Z*1, the *COG* of barbell position on the *Z-*axis is *Z*2, the weight of lifter is *M*1, and the weight of barbell is *M*2.

(3) $$\begin{array}{c} Z_{c}=\frac{\left(\text{Z}1\times M1+Z2\times M2\right)}{\left(M1+M2\right)}. \end{array}$$

### 2.3. Statistical Analyses

The homogeneity of variance and normal distribution assumptions were analyzed by Levene's tests and Kolmogorov-Smirnov, respectively. Using Box-whisker plot to test outliers in variables. The data comparison was analyzed by a paired-sample *t* test and calculated the linear variation with time of human and bar combination barycenter on *X-*axis using a linear regression equation. *P* < 0.05 indicates a significant difference between successful and failed snatch. The results of statistical analysis were obtained using the IBM SPSS 20.0 (SPSS Inc., Chicago, IL, USA).

The article "A Biomechanical Study on Failed Snatch Based on the Human and Bar Combination Barycenter" was published in 2022. Journal: Appl Bionics Biomech.

## 3. Results

### 3.1. Comparison of the Characteristics of “Near,” “Fast,” and “Low” Principles

Comparison the successful and failed snatch of the ten lifters, the characteristics of “Near,” “Fast,” and “Low” principles are shown in Table 2. There were no significant differences between success and failure in the minimum horizontal distance between the *COG* of barbell and human body during the barbell rising (*L*_Hmin_), in the maximal vertical rising velocity (*V*_max_), in the maximal vertical height (*H*_bmax_), in the vertical height of human body (*H*_bd5_) and barbell (*H*_b5_) at the end of *M*5, and in the vertical distance between the *COG* of barbell and human body at the end of *M*5 (*L*_Hz2_). Furthermore, there was no significant difference between success and failure in the maximum falling acceleration of the *COG* of human body (*a*_*f*_) (*t* = −1.189, *P* = 0.265). In the successful attempts, the *a*_*f*_ is 0.3938 m/s^2^ greater than that in unsuccessful attempts. However, it is worth noting that the *a*_*f*_ of eight lifters in successful and unsuccessful actions are greater than the acceleration of gravity (*g* = 9.8 m/s^2^), and the *a*_*f*_ of other two lifters are less than the acceleration of gravity. In addition, significant difference (*t* = 4.043, *P* = 0.01) could be found between success and failure in the vertical distance between the *COG* of barbell and human body at the end of *M*4 (*L*_Hz1_). The *L*_Hz1_ in successful attempts is 1.95 cm larger than that in unsuccessful actions.

### 3.2. Comparison of the Characteristics of Phases

In order to analyze the characteristics of snatch in more details, the snatch process is usually divided into several phases. In the present study, the snatch from start to the squat position was divided as six phases (Figure 2). Since the unsuccessful attempts all occur in the *M*6, the comparison of phase characteristics does not include the *M*6. The vertical displacement of each phase of barbell, the duration time, and the angles of the hip and knee joints at the end of each phase is chosen for analyzing. The comparison of the characteristics of phases between the successful and unsuccessful attempts is shown in Tables 3 and 4. In the present study, there was no significant difference between success and failure of the ten weightlifters in the vertical displacement and duration time of each phase, the angle of hip, and knee joints at the end of the six phases.

The article "A Biomechanical Study on Failed Snatch Based on the Human and Bar Combination Barycenter" was published in 2022. Journal: Appl Bionics Biomech.

### 3.3. Comparison of Human and Bar Combination Barycenter

The “combination barycenter” is derived from the calculation of the *COG* of combined objects in physics. The human and bar combination barycenter is to view the human body and barbell as a whole, the combination barycenter of the *COG* of body and barbell. Before calculating the human and bar combination barycenter, the data are unified firstly, and the 3-D coordinates are defined as *X*-, *Y*-, and *Z*-axis. Set the 3-D coordinates of the *COG* of barbell before the snatch to (0, 0, 0.225), and the corresponding 3-D coordinates of the *COG* of body are processed accordingly, so that the 3-D coordinates at the beginning of all attempts are consistent. The comparison of the human & bar combination barycenter between the successful and unsuccessful attempts on the *X*-, *Y*-, and *Z*-axis are shown in Figures 4–6.

The trajectory changes of the human and bar combination barycenter of the successful and unsuccessful attempts on the *X-*axis are shown in Figure 4. The displacement of human and bar combination barycenter of ten lifters all increase with time, and the slopes of successful snatch of all lifters are higher than that of unsuccessful snatch.  Figure 5 shows the trajectory changes of human and bar combination barycenter of successful and unsuccessful attempts on the *Y-*axis. The offsets of all lifters on the *Y-*axis are very small, and there is no obvious regular pattern.  Figure 6 shows the trajectory changes of the human and bar combination barycenter on the *Z-*axis. The trajectories of human and bar combination barycenter of successful and unsuccessful on the *Z-*axis show a trend of rising first and then decreasing, and the trajectories show a high degree of consistency.

In order to further study the characteristics of human and bar combination barycenter of successful and failed attempts, the present study intercepted the values of the human and bar combination barycenter on the *X-*axis at the characteristic pictures of each phase and calculated the variation of each phase and compared the difference of human and bar combination barycenter between successful and failed attempts on the *X-*axis. Secondly, this study used the method of calculating the cumulative variation to analyze the difference of the human and bar combination barycenter between the successful and unsuccessful actions on the *Y-* and *Z-*axis.

The article "A Biomechanical Study on Failed Snatch Based on the Human and Bar Combination Barycenter" was published in 2022. Journal: Appl Bionics Biomech.

Table 5 shows the results of displacement of the human and bar combination barycenter at the characteristic pictures of each phase and displacement change of each phase of successful and failed snatch on the *X-*axis. There are significant differences in the displacement of human and bar combination barycenter on the *X-*axis between successful and failed snatch at the end of *M*1, *M*2, *M*4, and *M*5 (*t* = 2.480, *P* < 0.05; *t* = 2.493, *P* < 0.05; *t* = 3.584, *P* < 0.05; *t* = 4.104, *P* < 0.05). There was no statistical difference at the beginning of *M*1 and the end of *M*3 (*t* = 1.429, *P* = 0.187; *t* = 2.152, *P* = 0.060). Since the change of the human and bar combination barycenter on the *X-*axis shows an upward trend, the change values were used to represent the variation of each phase. Significant differences were found in the variation of human and bar combination barycenter between successful and unsuccessful on the *X-*axis in the phase of *M*4 and *M*5 (*t* = 2.862, *P* < 0.05; *t* = 3.376, *P* < 0.05). In the other three phases, there was no significant difference between success and failure (*t* = 0.176, *P* = 0.864; *t* = 1.383, *P* = 0.200; *t* = 1.824, *P* = 0.102).

Since the change of human and bar combination barycenter fluctuates on the *Y-*axis and *Z-*axis, the cumulative variation in phase is used to analyze the characteristics of the successful and failed attempts (Table 6). Assuming that there *n* frames in each phase, the calculation formula of the cumulative variation (*Y*_*cn*_) of the human and bar combination barycenter on the *Y-*axis in this phase is as follows (the calculation of *Z*_*cn*_ and *Y*_*cn*_ is the same):

(4) $$\begin{array}{c} Y_{cn}=\left|Yc2-Yc1\right|+\left|Yc3-Yc2\right|\cdots +\left|Ycn-Yc\left(n-1\right)\right|. \end{array}$$

There is no significant difference (Table 6) in the cumulative variation of the human and bar combination barycenter on the *y-*axis at each phase between success and failure (*t* = 1.025, *P* = 0.332; *t* = −1.326, *P* = 0.217; *t* = 1.012, *P* = 0.338; *t* = −0.319, *P* = 0.757; *t* = −0.931, *P* = 0.376). And there is no significant difference in the cumulative variation of the human and bar combination barycenter on the *Z-*axis at each phase between success and failure (*t* = −0.496, *P* = 0.632; *t* = −1.556, *P* = 0.154; *t* = 1.275, *P* = 0.234; *t* = 1.433, *P* = 0.186; *t* = −1.112, *P* = 0.295).

### 3.4. Analysis of the Regression Equation of the Human and Bar Combination Barycenter on the *X-*Axis during the Phases of *M*4 and *M*5

Given that the differences of human and bar combination barycenter on the *X-*axis between successful and failed attempts mainly occur in the *M*4 and *M*5 phases, the present study established the regression equations of the displacement change of the human and bar combination barycenter on the *X-*axis with time in these two phases. Take time as the independent variable (*χ*) and the value of human & bar combination barycenter on the *X-*axis as the dependent variable (*y*). The regression equation model was used to establish a linear unitary regression equation for the success and failure in the phases of *M*4 and *M*5 (Table 7). The fitting degree of each linear regression equation model is represented by the *R*^2^ value (Table 8), and the *R*^2^ values of all regression equation models are greater than 0.85, indicating that the data is well fitted and linear. The *t*-test of all independent variables of the regression equation is less than 0.001, and the sample regression coefficient (the slope of the regression line) of successful linear regression equation of each athlete is greater than the failure.

The article "A Biomechanical Study on Failed Snatch Based on the Human and Bar Combination Barycenter" was published in 2022. Journal: Appl Bionics Biomech.

## 4. Discussion

### 4.1. Analysis of the “Near,” “Fast,” and “Low” Principles and the Parameters in Phases

In the present study, the snatch can be divided into two parts: the first part is from the moment of snatch start to the barbell's maximum vertical velocity; the second part is from the beginning of the barbell's inertial rise to the athlete's squatting and receiving the barbell. The first part can be divided into three phases: knee extension phase (*M*1), knee flexion phase (*M*2), and force phase (*M*3). This part is mainly for athletes to lift the barbell, give the barbell an upward force, so that the barbell can gain a certain speed and height and obtain the most appropriate initial velocity (*V*_max_) at the end of this part. The 2^nd^ part can be divided into three stages: the inertial ascent stage (*M*4), the squat support stage (*M*5), and the support completion stage (*M*6). The second part mainly uses the speed obtained in the first part to make the barbell continue to rise inertially, while relying on “swing arms and turning wrists” [29] which make the barbell continue to gain a certain speed during the inertial ascent. At the same time, the reaction force of the barbell acts on the human body to make lifter obtain greater downward acceleration, so as to quickly squat to support and receive barbell [30, 31].

Previous studies [10, 32–35] pointed out that insufficient knee flexion in the knee flexion phase is one of the important factors leading to the failure of snatch. At the knee flexion phase, athletes need to actively extend the hip joint and fully flex the knee joint. On the contrary, that is, knee joint is not fully flexed, and the extension of the hip joint is limited. The present study compared the characteristics of the successful and failed attempts of ten athletes. In the first part, the minimum horizontal distance between the *COG* of the human body and barbell, the barbell's maximum vertical velocity, the time parameters, space parameters, and the joints angle are all compared. There is no statistical difference, which showed that there was no obvious difference between the success and failure in the first part, which is consistent with related research [4, 15]. Although all parameters were not statistically different, some parameters are still worthy of our attention because they are very important for technical actions [36, 37]. For instance, the average value of the knee angle of the successful attempts is 6.99° smaller than that of failed attempts at the end of the knee flexion phase, and the maximum vertical velocity of successful attempts is 0.0847 m/s greater than that of failure. Insufficient knee flexion will affect the secondary force and will inevitably affect the maximum velocity of the barbell. It may be a potential factor for snatch failure. However, in this study, due to research limitations, it cannot be confirmed that the direct cause of snatch failure is insufficient knee flexion.

The article "A Biomechanical Study on Failed Snatch Based on the Human and Bar Combination Barycenter" was published in 2022. Journal: Appl Bionics Biomech.

The study of Wang and Liu [18] showed that the maximum vertical distance between the *COG* of body and barbell is not enough to form a favorable support posture, which may be the main reason for the failed snatch. The studies of Gourgoulis et al. [4, 15] pointed out that there is no significant difference in the temporal and spatial characteristics between successful and failed snatch. In our study, the successful and failed attempts of ten athletes were compared. In addition to the significant difference in the vertical distance between the *COG* of barbell and human body at the end of the inertial ascent stage (*M*4) in the second part, there are no significant differences in the vertical acceleration of body, time parameters, spatial parameters, and joints angle. Since there is no significant difference in the barbell's maximal vertical height at the end of the inertial ascent stage (*M*4) between the successful and failed attempts, the average difference is only 0.049 cm. However, the vertical distance between the *COG* of body and barbell is different at the end of the inertial ascent stage (*M*4), the *L*_Hz1_ of successful snatch is 1.95 cm larger than that of failed snatch, which indicates that the falling velocity of the *COG* of body of successful attempts is higher than that of failed attempts in the inertial ascent stage (*M*4). At the same time, the average hip and knee angles of the successful attempts are less than those of the failed attempts at the end of the squat support stage (*M*5). There is no significant difference in the vertical height of *COG* of human body, the vertical height of barbell, and the vertical distance between the *COG* of human body and barbell at the end of the squat support stage (*M*5). Based on these, the insufficient support space may be one of the reasons for failure which pointed out in related study [18], and the conclusion lack sufficient evidence. The results of the present study are basically consistent with the results of previous studies [4, 15].

The article "A Biomechanical Study on Failed Snatch Based on the Human and Bar Combination Barycenter" was published in 2022. Journal: Appl Bionics Biomech.

### 4.2. Analysis of the Human and Bar Combination Barycenter

The human and bar combination barycenter is the *COG* formed by the combination of the *COG* of barbell and *COG* of human body. The changes of the human and bar combination barycenter is affected by the change of the *COG* of barbell and/or *COG* of human body. The change of the human and bar combination barycenter on the *Y-*axis indicates that the left and right deviation of the *COG* of barbell and human body in the snatch. The smaller the cumulative change in each phase, the smaller offset of the *COG* of barbell and human body in this stage, and more stable snatch technique. The results of the present study showed that the human and bar combination barycenter on the *Y-*axis of successful attempts is greater than the failure in *M*1 and *M*3, but there is no significant difference (Table 6). There is no significant difference in the cumulative change of the human and bar combination barycenter on the *Z-*axis, and Figure 6 shows that the change of the human and bar combination barycenter for successful and failed snatches tends to be consistent.

Compared the changes of the human and bar combination barycenter on the *X-*axis between the successful and failed attempts, it was found that the values of the end of knee extension phase (*M*1), the knee flexion phase (*M*2), the inertial ascent stage (*M*4), and the squat support stage (*M*5) are statistically different. And the changes in the inertial ascent stage (*M*4) and in the squat support stage (*M*5) are also statistically different, all the successful attempts are greater than the failed attempts. The average value of human and bar combination barycenter at the end of knee extension phase (*M*1) of successful attempts is 0.4816 cm larger than the failed attempts. The average value of human and bar combination barycenter at the end of knee flexion phase (*M*2) of successful attempts is 0.8955 cm larger than the failed attempts. The average value of human and bar combination barycenter at the end of the inertial ascent stage (*M*4) of successful attempts is 2.3362 cm larger than the failed attempts. The average value of human and bar combination barycenter at the end of the squat support stage (*M*5) of successful attempts is 2.729 cm larger than the failed attempts. The variation of human and bar combination barycenter in the inertial ascent stage (*M*4) of successful attempts is 1.2718 cm larger than the failed attempts. And the variation of human and bar combination barycenter in the squat support stage (*M*5) of successful attempts is 0.4676 cm larger than the failed attempts. These indicate that the key problems of failed snatch are caused by the insufficient increase of human and bar combination barycenter on the *X-*axis during the inertial ascent stage (*M*4) and the squat support stage (*M*5).

The article "A Biomechanical Study on Failed Snatch Based on the Human and Bar Combination Barycenter" was published in 2022. Journal: Appl Bionics Biomech.

In the present study, the unitary regression equations were established from the beginning of the inertial ascent stage (*M*4) to the end of the squat support stage (*M*5) of the success and failure of ten athletes. It can be seen from Table 7 that the slope of the regression line for success is greater than that for failure.  Figure 7 shows the changes of *COG* of barbell, *COG* of body, and human and bar combination barycenter on the *X-*axis during the entire snatch process. It is easy to find that the gap of the human and bar combination barycenter between successful and failed attempts is getting bigger and bigger over time; especially, after the beginning of the inertial ascent stage, the slope of the human and bar combination barycenter of successful is obviously higher than that of the failure. The trajectory of the *COG* of barbell shows a trend of falling first and then rising from this stage, while the trajectory of *COG* of body shows the opposite trend of rising first and then failing. If weightlifters want to maintain the continuous growth of the human and bar combination barycenter, they need to reduce the downward trend of the *COG* of barbell and increase the growth trend of the *COG* of body.

From the perspective of technical performance, the barbell obtained the maximum vertical velocity after the force phase (*M*3) is over. By now, the *COG* of body drops rapidly, with the elbow joint as the center of the circle, and the forearm as the radius to swing the barbell to continue rising. Previous research [29] pointed out that since the barbell moves in an arc form during the inertial ascent stage, the force on the barbell can be decomposed into a vertical upward force *F*1 and a positive *X-*axis force *F*2. *F*1 raises the barbell to the maximum height, and *F*2 brings the barbell close to the body and reaches the support position. If *F*2 is too large, the *COG* of barbell will move backward and cause the barbell to fall behind, and if *F*2 is too small, it will cause the *COG* of barbell to move forward and cause the barbell to fall forward. The power of *F*1 mainly comes from the “swing arms and turning wrists”, while the power of *F*2 comes from the proper upper body reclining at the end the force phase (*M*3). At this stage, the *COG* of human body relies on the reaction force of the barbell and hip and knee flexion to actively descend. It is worth noting that some studies have pointed out that the falling acceleration of human body of elite weightlifters should be greater than the acceleration of gravity (*g* = 9.8 m/s^2^). In the present study, the maximum acceleration of human body in eight weightlifters is greater than the acceleration of gravity, which shows that the squatting and supporting technique of the two other lifters still need to be improved.

The article "A Biomechanical Study on Failed Snatch Based on the Human and Bar Combination Barycenter" was published in 2022. Journal: Appl Bionics Biomech.

The present study believes that a probable cause of the failure is that the human and bar combination barycenter does not reach the specified position, and the reason is insufficient backward leaning of torso at the end of the force phase (*M*3). The research of Gourgoulis et al. [4, 15] showed that the difference of the resultant acceleration on the vector direction and the instability of the force direction during the knee extension phase (*M*1) are the main reasons for the failure of snatch. The probable reasons for the difference may be that multiple categories of lifters (69 kg, 77 kg, and 85 kg) were selected in literatures, and individuals are quite different. Furthermore, they did not distinguish the type of failure (the barbell falls forward or backward). In the present study, all the unsuccessful attempts are forward falling.

In summary, compared the characteristics of successful and failed snatch, it is concluded that the probable cause of the failure is that the position of the human and bar combination barycenter on the *X-*axis is more forward than the position of the successful attempts at the end of the inertial ascent stage (*M*4) and the squat support stage (*M*5). The reasons are that the upper body does not lean back properly at the end of the force phase (*M*3) and the shoulder, waist, and back muscles are not used to give proper force to barbell, which leads to the growth of the human and bar combination barycenter on the *X-*axis is insufficient during the inertial ascent stage (*M*4) and the squat support stage (*M*5), and result in failure of *COG* of barbell to reach the proper position and finally causing the snatch failure. In addition, insufficient knee flexion in the knee flexion phase (*M*2) leads to insufficient secondary force, which causes the maximum vertical velocity of barbell to be too low, and it may also be an indirect factor that causes the snatch failure, because the insufficient maximum vertical velocity may cause the lifters to use more power for barbell rising and reduce the force on the positive direction of the *X-*axis during inertial ascent stage (*M*4), which indirectly leads to the failure of the snatch. Therefore, in the present study, the effectiveness of human and bar combination barycenter in judging the successful and failed attempts of elite weightlifters has been verified.

The article "A Biomechanical Study on Failed Snatch Based on the Human and Bar Combination Barycenter" was published in 2022. Journal: Appl Bionics Biomech.

### 4.3. Limitations

In order to avoid the influence of technical differences between weightlifting categories, the present study only selected the men's 73 kg category snatch competition in recent years. The relatively small number of research samples is one of the limitations of this study. In addition, the present study only discussed the factors for the failure of the barbell to fall forward, and whether it is also effective for the backward drop still needs further verification. Furthermore, the video was obtained under competitive conditions only using two cameras. It is inevitable that the body joints, such as the knee joint, are hidden by local limbs or not visible on side camera when video digitizing. Under this circumstance, the method of zooming in the local joints we used makes the joints of human body more clearly, which is helpful for the accuracy of the data. However, there are still some limitations compared with the multicamera method.

## 5. Conclusions

The present study compared the successful and failed techniques of snatch of elite lifters and analyzed the characteristics of “Near,” “Fast,” and “Low” principles, the parameters in phases, and the parameters of human and bar combination barycenter. And we established the regression equation of the human and bar combination barycenter on the *X-*axis during the inertial ascent stage (*M*4) and the squat support stage (*M*5). And we found the effectiveness of the human and bar combination barycenter in judging success and failure snatch. The main conclusions are as follows:

1. A probable cause of the failed snatch is that the displacement of human and bar combination barycenter on the *X-*axis is not enough to reach the position for supporting barbell during the inertial ascent stage (*M*4) and the squat support stage (*M*5). The reason is that the strength of reclining of t torso at the end of the force phase (*M*3) is insufficient, so it is reminded that weightlifters who often fall forward in snatch should strengthen reclining exercises
2. Insufficient knee flexion during the knee flexion stage (*M*2) leads to a lower maximal vertical velocity of barbell and difference of vertical distance between the *COG* of human body and barbell at the end of the inertial ascent stage (*M*4), which may be an indirect factor leading to the failure of snatch
3. The cumulative variation of human and bar combination barycenter on the *X-*axis can effectively determine the technical characteristics between the success and failure of elite weightlifters in snatch

The article "A Biomechanical Study on Failed Snatch Based on the Human and Bar Combination Barycenter" was published in 2022. Journal: Appl Bionics Biomech.

## Figures and Tables

**Figure 1:** Experimental design and 3-D coordinate system.

**Figure 2:** The feature pictures of each phase of snatch.

**Figure 3:** Seventeen key points on the human body and barbell manually digitized.

**Figure 4:** The trajectories of the human and bar combination barycenter of successful and unsuccessful snatch on the *X-*axis.

**Figure 5:** The trajectories of the human and bar combination barycenter of successful and unsuccessful snatch on the *Y-*axis.

**Figure 6:** The trajectories of the human and bar combination barycenter of successful and unsuccessful snatch on the *Z-*axis.

**Figure 7:** Successful and unsuccessful trajectories of the *COG* of barbell and body and human and bar combination barycenter on the *X-*axis.

**Table 1:** Information of subjects (*n* = 10).

Subjects	Body mass (kg)	Height (m)	Heaviest successful weight (kg)	Heaviest unsuccessful weight (kg)
1	72.88	1.70	155	150
2	72.56	1.71	155	146
3	73.00	1.68	158	154
4	72.79	1.70	146	140
5	72.90	1.68	146	144
6	72.55	1.71	161	156
7	73.00	1.74	148	145
8	72.39	1.69	156	151
9	72.92	1.70	150	148
10	72.63	1.65	144	140

**Table 2:** Comparative analysis of the parameters of “Near,” “Fast,” and “Low” principles.

	Successful	Unsuccessful
*L*_Hmin_ (m)	0.04192 ± 0.0158	0.0431 ± 0.0163
*V*_max_ (m/s)	1.6984 ± 0.1421	1.6137 ± 0.16342
*H*_bmax_ (m)	1.1791 ± 0.03618	1.1840 ± 0.11316
*a*_*f*_ (m/s^2^)	−13.0760 ± 4.6054	−12.6822 ± 4.4197
*L*_Hz1_ (m)	0.5152 ± 0.0354	0.4957 ± 0.0386^∗^
*H*_b5_ (m)	1.1193 ± 0.0421	1.1083 ± 0.0349
*H*_bd5_ (m)	0.5236 ± 0.0232	0.5180 ± 0.0321
*L*_Hz2_ (m)	0.5912 ± 0.0467	0.5914 ± 0.0164

^∗^Statistically significant difference (*P* < 0.05).

**Table 3:** Vertical displacement of barbell and time duration of each phase of the successful and unsuccessful snatch.

	Vertical displacement of each phase (m)		Duration of each phase (s)	
	Successful	Unsuccessful	Successful	Unsuccessful
*M*1	0.5584 ± 0.0839	0.5533 ± 0.0674	0.454 ± 0.049	0.458 ± 0.0537
*M*2	0.1271 ± 0.0389	0.1312 ± 0.0508	0.290 ± 0.2354	0.300 ± 0.2400
*M*3	0.2610 ± 0.0541	0.2566 ± 0.0516	0.416 ± 0.2819	0.409 ± 0.2837
*M*4	0.2889 ± 0.0278	0.2784 ± 0.0189	0.552 ± 0.3821	0.546 ± 0.3737
*M*5	0.0593 ± 0.0054	0.0648 ± 0.0117	0.532 ± 0.4896	0.536 ± 0.4903

The article "A Biomechanical Study on Failed Snatch Based on the Human and Bar Combination Barycenter" was published in 2022. Journal: Appl Bionics Biomech.

**Table 4:** Angles of hip and knee joints at the end of each phase of successful and unsuccessful snatch.

	Knee angel (degree)		Hip angle (degree)	
	Successful	Unsuccessful	Successful	Unsuccessful
*M*1	121.85 ± 11.42	124.24 ± 9.93	85.02 ± 5.63	88.87 ± 14.27
*M*2	111.9 ± 6.47	118.89 ± 9.22	111.18 ± 7.75	112.22 ± 7.39
*M*3	153.13 ± 9.22	151.84 ± 7.88	144.68 ± 19.58	152.64 ± 6.54
*M*4	68.47 ± 8.38	68.72 ± 9.37	99.08 ± 20.43	101.67 ± 18.78
*M*5	44.71 ± 6.2	45.29 ± 10.34	52.38 ± 11.62	58.72 ± 16.45

**Table 5:** The displacement of the human and bar combination barycenter at the characteristic pictures and the variation of each phase of successful and failed snatch on the *X-*axis (cm).

	Value of characteristic pictures			Variation of phases	
	Successful	Unsuccessful		Successful	Unsuccessful
*a*	1.7431 ± 1.1772	1.5077 ± 1.1016			
*b*	4.5164 ± 2.6399	4.0348 ± 2.6847^∗^	*M*1	2.9789 ± 1.4836	2.9305 ± 1.9815
*c*	5.498 ± 3.2521	4.6025 ± 2.9853^∗^	*M*2	1.8293 ± 2.5905	0.716 ± 0.3614
*d*	6.7040 ± 3.1200	5.7138 ± 3.4461	*M*3	1.5435 ± 0.4132	1.2525 ± 0.6647
*e*	9.9856 ± 5.6563	7.6494 ± 4.7551^∗^	*M*4	3.3174 ± 2.5498	2.0456 ± 1.2762^∗^
*f*	10.9535 ± 6.2216	8.2245 ± 5.4097^∗^	*M*5	1.3129 ± 1.1732	0.8453 ± 0.9844^∗^

^∗^Statistically significant difference (*P* < 0.05).

**Table 6:** The cumulative change of the human and bar combination barycenter of successful and failed snatch on the *Y-*axis and *Z-*axis.

	*Y-*axis		*Z-*axis	
	Successful	Unsuccessful	Successful	Unsuccessful
*M*1	2.3924 ± 1.7699	2.119 ± 1.6302	25.7886 ± 4.0861	26.2975 ± 3.642
*M*2	0.3357 ± 0.1692	0.5692 ± 0.5474	8.7441 ± 4.8083	11.4343 ± 4.0532
*M*3	1.2283 ± 0.7987	1.0141 ± 0.8591	23.0791 ± 5.1511	20.8446 ± 4.0949
*M*4	1.6672 ± 1.3182	1.7646 ± 1.1674	14.9653 ± 2.5195	13.9429 ± 2.1093
*M*5	0.7373 ± 0.3157	0.9771 ± 0.8159	7.5426 ± 1.8076	8.1324 ± 1.3437

**Table 7:** Linear regression equation of variation trend of the human and bar combination barycenter on the *X-*axis.

Subjects	Successful	Unsuccessful
1	*y* = −0.006 + 0.138*χ*	*y* = −0.009 + 0.71*χ*
2	*y* = −0.042 + 0.153*χ*	*y* = −0.017 + 0.098*χ*
3	*y* = −0.078 + 0.133*χ*	*y* = −0.012 + 0.099*χ*
4	*y* = 0.005 + 0.066*χ*	*y* = 0.029 + 0.019*χ*
5	*y* = 0.056 + 0.041*χ*	*y* = 0.071 + 0.021*χ*
6	*y* = −0.119 + 0.322*χ*	*y* = −0.034 + 0.186*χ*
7	*y* = −0.050 + 0.205*χ*	*y* = −0.019 + 0.118*χ*
8	*y* = 0.022 + 0.038*χ*	*y* = 0.025 + 0.028*χ*
9	*y* = 0.001 + 0.042*χ*	*y* = −0.018 + 0.0272*χ*
10	*y* = 0.015 + 0.037*χ*	*y* = −0.013 + 0.010*χ*

**Table 8:** *R* ^2^ value of linear regression equation of variation trend of the human and bar combination barycenter on the *X*-axis.

Subjects	Successful		Unsuccessful	
	*R* ^2^	*P* value	*R* ^2^	*P* value
1	0.972	≤0.001	0.983	≤0.001
2	0.987	≤0.001	0.952	≤0.001
3	0.969	≤0.001	0.976	≤0.001
4	0.956	≤0.001	0.958	≤0.001
5	0.942	≤0.001	0.891	≤0.001
6	0.941	≤0.001	0.968	≤0.001
7	0.934	≤0.001	0.978	≤0.001
8	0.892	≤0.001	0.877	≤0.001
9	0.883	≤0.001	0.852	≤0.001
10	0.855	≤0.001	0.857	≤0.001

The article "A Biomechanical Study on Failed Snatch Based on the Human and Bar Combination Barycenter" was published in 2022. Journal: Appl Bionics Biomech.

## Data Availability

The data of the present study that support the findings are available from the corresponding author upon reasonable request.
